# MiR-140-5p suppresses retinoblastoma cell growth via inhibiting c-Met/AKT/mTOR pathway

**DOI:** 10.1042/BSR20180776

**Published:** 2018-11-30

**Authors:** Yujun Liao, Xiaolong Yin, Yan Deng, Xiaowei Peng

**Affiliations:** Department of Pediatric Ophthalmology, The Second Affiliated Hospital of Nanchang University, Nanchang 330000, China

**Keywords:** c-Met/AKT/mTOR signaling pathway, MiR-140-5p, retinoblastoma, tumorigenesis

## Abstract

MiR-140-5p is low expression and acts as a tumor suppressor in various types of human cancers. However, the potential role of miR-140-5p in retinoblastoma (RB) remains unknown. In the present study, we performed the miRNA microarray analysis to investigate whether miRNAs expression are associated with RB tumorigenesis in RB tissues. We found that a large set of miRNAs were ectopic expressions and miR-140-5p is most significantly down-regulated in human RB tissues compared with normal retinas. In addition, low miR-140-5p expression is associated with clinicopathological features (differentiation, invasion, T classification, N classification, cTNM stage, and largest tumor base) and poor survival in RB patients. Furthermore, our results showed that overexpression of miR-140-5p suppresses proliferation and induces apoptosis and cell cycle arrest in RB cell. Meanwhile, we confirmed that c-Met is the functional target of miR-140-5p in RB cell, and miR-140-5p expression is negatively correlated with c-Met in RB tissues. We also found that inhibition of c-Met also suppresses proliferation and induces apoptosis and cell cycle arrest in RB cell. Interestingly, c-Met can rescue the suppressive effects of miR-140-5p on RB cell growth and cell cycle arrest. More importantly, our findings indicated that miR-140-5p may inhibit cell growth via blocking c-Met/AKT/mTOR signaling pathway. Collectively, these results suggested that miR-140-5p might be a potential biomarker and target in the diagnosis and treatment of RB.

## Introduction

Retinoblastoma (RB) is the most common childhood malignancy with 1000 newly diagnosed cases annually in China [1]. RB affects the eyes of children at a very young age and accounts for 5% of blindness in children [2]. Many patients with RB have high mortality rate due to their failure to be diagnosed during the early stage, especially in developing countries [3]. Currently, chemotherapy is often used to reduce mortality and improve the prognosis of patients with RB [4]. However, it has been regarded as one of the deadliest forms of cancer due to its limited sensitivity to chemotherapy [5]. Therefore, there is an urgent need to search for useful biomarkers and explore novel targets in both clinical diagnosis and treatment for RB.

MicroRNAs (miRNAs), are a family of short, noncoding RNA molecules consisting of 19–25 nts, which act as negative post-transcriptional regulators of target genes [6]. miRNAs have been identified to be involved in many physiological and pathological processes, including proliferation, death, differentiation, and metabolism [7]. Growing evidence revealed that miRNAs are dysregulated and play important roles in a variety of cancers via functioning as potent oncogenes or tumor suppressor genes [8]. Recent studies demonstrated that the ectopic expression of miRNAs can modulate cell proliferation, apoptosis, and metastasis in RB [9–11]. Mu et al. [12] reported that miR-let-7 is down-regulated in RB and may be associated with tumorigenesis and progression of RB. Plasma miR-320, miR-let–7e, and miR-21 were identified to serve as novel potential biomarkers for the diagnosis of RB [13]. Recently, miR-140-5p has been reported to be down-regulated and act as a tumor suppressor in various human cancers, including ovarian cancer [14], non-small cell lung cancer [15], colorectal cancer [16], and gastric cancer [13]. However, the molecular mechanism underlying the role of miR-140-5p in the development of RB remains unclear.

In the present study, we identified miRNA expression profiles in RB tumorigenesis and investigated the molecular mechanism underlying the biological function of miRNAs in the development of RB. Our results showed that miR-140-5p is down-regulated in RB tissues and its expression predicts poor prognosis in RB. Furthermore, our findings uncovered that miR-140-5p suppresses proliferation and induces apoptosis and cell cycle arrest through blocking c-Met/AKT/mTOR signaling pathway, and suggested the potential value of miR-140-5p in RB clinical diagnosis and treatment.

## Materials and methods

### Patients and tissue samples

A total of 50 RB tissues and 8 normal retinas were obtained from the Department of Pediatric Ophthalmology, the Second Affiliated Hospital of Nanchang University from February 2013 to November 2016. Tissues were collected from patients who had not received radiotherapy or chemotherapy prior to surgical resection. The clinicopathological features of RB patients are summarized in Table 1. All 50 RB patients were identified histopathologically and staged according to the American Joint Commission for Cancer (AJCC) staging system. The normal retinas were collected from eight patients who had died of conditions other than ophthalmologic diseases in the Department of Pediatric Ophthalmology, the Second Affiliated Hospital of Nanchang University. All patients provided written informed consent for the use of human specimens for clinical research. The present study was approved by the institute research ethics committee of the Second Affiliated Hospital of Nanchang University.

**Table 1:** Correlation between miR-140-5p and clinicopathological features in RB patients

Clinical parameters	All cases, *n*=50	miR-140-5p expression		*P*-value
		High (22)	Low (28)	
Gender				0.615
Male	23	11	12	
Female	27	11	16	
Age (years)				0.477
≥5	9	3	6	
<5	41	19	22	
Tumor enucleated location				0.802
Right	26	11	15	
Left	24	11	13	
Differentiation				0.035*
Well and moderate	28	16	12	
Poor	22	6	16	
Invasion				0.033*
Noninvasive	19	12	7	
Invasive	31	10	21	
T classification				0.061
T1 + T2	29	16	13	
T3 + T4	21	6	15	
N classification				0.015*
N0	20	13	7	
N1 + N2	30	9	21	
cTNM stage				0.013*
I + II	12	9	3	
III + IV	38	13	25	
Largest tumor base (mm)				0.014*
≥15	16	3	13	
<15	34	19	15	
Tumor thickness (mm)				0.254
≥10	25	13	12	
<10	25	9	16	

* *P*<0.05.

### Cell culture

The human RB cell lines Y79 (HTB-18), Weri-Rb1 (HTB-169), SO-Rb50, and HXO-RB44 and human retinal pigment epithelium (RPE) cell were purchased from the American Type Culture Collection (ATCC, Rockville, MD, U.S.A.). All the cells were maintained in RPMI 1640 (Life Technologies, Grand Island, NY, U.S.A.) supplemented with 10% FBS (Sigma), 100 IU/ml penicillin (Life Technologies), and 100 mg/ml streptomycin (Life Technologies), at 37°C in a humidified atmosphere containing 5% CO_2_ (Thermo).

### Cell transfection

The specific miR-140-5p mimics/inhibitor and corresponding negative control (NC), as well as specific siRNA for c-Met (si-c-Met) and si-Scramble were designed and purchased from GenePharma Co., Ltd (Shanghai, China). The target siRNA sequence for c-Met was: si-c-Met, 5′-CACAACAGTGTGGACCACAAGAGAT-3′; si-Scramble, 5′-CACTGACGGTGACCAGAACAAAGAT-3′. These oligo fragments were transfected into cells using Lipofectamine 2000 (Invitrogen, Carlsbad, CA, U.S.A.) according to the manufacturer’s instructions. At 48 h after transfection, cells were collected for further analysis.

### miRNA microarray analysis

miRNA microarray analysis was conducted to determine miRNA expression profiles in tissue samples. Total RNAs were extracted by TRIzol reagent (Invitrogen, Carlsbad, CA, U.S.A.), and the miRNA fraction was further purified using a mirVana miRNA isolation kit (Ambion, Austin, TX) according to manufacturer’s protocol. The isolated miRNAs were labeled with Hy3 using the miRCURY array labeling kit (Exiqon, Vedbaek, Denmark) and hybridized with miRCURY locked nucleic acid (LNA) microRNA arrays (v8.0; Exiqon). Microarray images were obtained using a Genepix 4000B scanner (Axon Instruments, Foster City, CA, U.S.A.) and analyzed with Genepix Pro 6.0 software (Axon Instruments).

### Quantitative real-time PCR

Total RNA from tissues and cells were isolated using TRIzol reagent (Invitrogen, Carlsbad, CA, U.S.A.) according to the manufacturer’s instructions. The c-Met and miRNA were reverse transcribed with TaqMan Gene Expression Assays kit and TaqMan MicroRNA Reverse Transcription kit (Applied Biosystems, Thermo Fisher Scientific, CA, U.S.A.), respectively. Quantitative RT-PCR reactions were performed using 7500 real-time PCR system (Bio-Rad, Hercules, CA, U.S.A.) according to standard instructions. The expression of miR-140-5p and c-Met in tissues and cells were normalized to the expression of U6 and GAPDH, respectively. The relative quantitation (2^−ΔΔ*C*^_t_) method was used to calculate data, and experiments were performed in triplicate.

### Cell Counting Kit-8 assay

The cells proliferation was evaluated using the Cell Counting Kit-8 (CCK-8) assay according to the manufacturer’s instructions [17]. The RB cells Y79 and Weri-Rb1 were transfected with miR-140-5p mimics or mimics NC, and cells were seeded in 96-well plate at a density (5 × 10^4^ cells/well) in 100-μl DMEM medium supplemented with 10% FBS. After 48 h incubation, CCK-8 reagent (10 μl) was added to each well and continuously cultured for 1 h in 5% CO_2_ (Thermo). The absorbance rates at 450 nm were measured using Microplate Reader (Bio-Rad, U.S.A.). Each experiment was performed independently at least three times.

### Apoptosis analysis

The cell apoptosis was determined by the flow cytometry analysis. The cells (1 × 10^6^) were seeded into six-well plates and were incubated at 37°C in a humidified chamber containing 5% CO_2_ for 48 h after transfection with miR-140-5p mimics or mimics NC. The cells then were harvested and washed twice with cold PBS, and were fixed with 70% cold ethanol at 4°C overnight. Subsequently, they were resuspended in binding buffer and stained with 5 μl of AnnexinV-FITC and 1 μl of propidium iodide (PI, 50 μg/ml) (BD Biosciences). Each experiment was repeated at least three times.

### Cell cycle analysis

The RB cells were seeded into six-well plates at a concentration of 5 × 10^4^ cells/well, and were transfected with miR-140-5p mimics or mimics NC. For flow cytometric analysis (FACSCalibur, BD Biosciences), the cells were prepared by using the BD Cycletest™ Plus DNA Reagent Kit (BD Biosciences) according to manufacturer’s instructions. The G_0_/G_1_ and G_2_/M ratios were determined using analysis software (Cell Quest, BD Biosciences).

### Luciferase assay

The miR-140-5p mimics/inhibitor and corresponding NC were obtained from GenePharma (Shanghai, China). The potential binding site between c-Met and miR-140-5p was searched using TargetScan (Figure 3A). The human c-Met 3′-UTR with wild-type (wt) and mutant (mut) containing the putative binding site of miR-140-5p were constructed (Figure 3B) and then were cloned into a pMIR-REPORT luciferase reporter vector (Ambion, U.S.A.). Site-directed mutagenesis of the miR-140-5p target-site in the c-Met 3′-UTR was performed using a QuikChange Kit (Qiagen). For the luciferase assay, the Y79 cells were cultured in 96-well plates and co-transfected with 400 ng of either pMIR-c-Met-3′-UTR or pMIR-c-Met-mut-3′-UTR, and 50 ng of miR-98 mimic/inhibitor or corresponding NC using Lipofectamine 2000 reagent (Invitrogen). Forty-eight hours after transfection, the relative firefly luciferase activity normalized with *Renilla* luciferase was measured using the Dual-Light luminescent reporter gene assay (Applied Biosystems).

### Western blot analysis

The cells were lysed as described previously [18]. The protein concentration was quantitated using BCA protein assay kit (Pierce, Rockford, IL). The protein (60 μg) sample was then separated by SDS/PAGE (10% gel) (Sigma–Aldrich, St. Louis, MO) and transferred to PVDF membranes (Millipore, Germany). The membrane was blocked with 5% skimmed milk at room temperature for 1 h, and incubated with primary antibodies against c-Met, p-Met, Met, p-KAT, KAT, p-mTOR, mTOR, p-s6, or s6 at 4°C overnight. These antibodies for the above-mentioned proteins were obtained from Santa Cruz Biotechnology (Santa Cruz Biotechnology, Santa Cruz, CA, U.S.A.). β-actin (Sigma, St. Louis, MO, U.S.A.) served as an internal control. Horseradish peroxidase–conjugated (HRP) antibodies (Santa Cruz Biotechnology, Santa Cruz, CA, U.S.A.) were used as the secondary antibodies. The signals were visualized using a chemiluminescence HRP Substrate (Millipore) and autoradiography. The band intensity was quantitated using alpha Imager software (Alpha Innotech Corporation, San Leandro, CA).

### Immunohistochemistry

Immunohistochemistry (IHC) was performed as previously described [2]. Anti-c-Met primary antibody was purchased from Santa Cruz Biotechnology (Santa Cruz, CA, U.S.A.). The immunostaining was visualized with diaminobenzidine (DAB; Sigma) for 3 min, and analyzed under a light microscope.

### Statistical analysis

All statistical analyses were performed using SPSS software (version 18.0; SPSS, Chicago, IL, U.S.A.). Experiments were conducted in triplicate and data were presented as the mean ± S.D. Differences between multiple groups were analyzed by one-way ANOVA with Tukey’s post-hoc test, and the means of two groups were analyzed by Student’s *t*test. *P*-value of <0.05 was defined significant and <0.01 was defined very significant. The survival analysis was determined using the Kaplan–Meier method.

## Results

### miR-140-5p is down-regulated in RB tissues and cells and is associated with poor patient survival rate

To investigate whether miRNAs expressions are associated with RB tumorigenesis, we performed the miRNA microarray analysis to identify the miRNA expression profiles in RB tissues and normal retinas. We found that a large set of miRNAs were ectopic expressions and miR-140-5p is most significantly down-regulated in human RB tissues compared with normal retinas (Figure 1A). To further verify these results, the qRT-PCR was used to measure the miR-140-5p level in RB tissues (*n*=50) and normal retinas (*n*=8). Consistent with miRNA microarray data, the expression level of miR-140-5p in RB tissues is obviously lower than that in normal retinas (*P*<0.01; Figure 1B). Moreover, miR-140-5p down-regulation is confirmed in the human RB cell lines Y79, Weri-Rb1, SO-Rb50, and HXO-RB44 using qRT-PCR (*P*<0.01; Figure 1C). To explore the correlation between miR-140-5p level and clinicopathological features in RB, the miR-140-5p expressions in RB tissues were divided into two groups according to its expression levels of miR-140-5p using its median as a cut-off, including the high miR-140-5p group (*n*=22) and the low miR-140-5p group (*n*=28). Our results indicated that low expression of miR-140-5p dramatically correlated with differentiation (*P*=0.035), invasion (*P*=0.033), T classification (*P*=0.061), N classification (*P*=0.015), cTNM stage (*P*=0.013), and largest tumor base (mm) (*P*=0.014), but no significant correlation was observed between miR-140-5p expressions and the patients’ gender, age, or tumor thickness (mm) (Table 1). To explore the correlation between miR-140-5p expression and RB patients’ prognosis, the Kaplan–Meier survival analysis was used to plot RB curves. The results showed that patients with low miR-140-5p expression (*n*=28) had significantly poorer overall survival rate compared with those with high miR-140-5p expression (*n*=22) (*P*=0.0133; Figure 1D). Collectively, these results demonstrated that miR-140-5p is down-regulated in RB tissues and low miR-140-5p level predicts poor prognosis in RB, suggesting miR-140-5p may act as a novel biomarker in the clinical diagnosis of RB.

**Figure 1:** miR-140-5p is down-regulated in human RB tissues and cells (**A**) The miRNA expression profiles were identified in RB tissues and normal retinas using the microarray analysis. Red or green color separately shows high or low expression in the heatmap. (**B**) The qPCR analysis was used to measure the relative expression of miR-140-5p in tumor tissues (*n*=50) and normal tissues (*n*=8). (**C**) The miR-140-5p expression was measured by qPCR analysis in the human RB cell lines Y79, Weri-Rb1, SO-Rb50, and HXO-RB44 and human RPE cell. (**D**) The Kaplan–Meier overall survival rate curve for RB patients (*n*=50) with low and high miR-140-5p expression levels (*P*=0.0133). Data were presented as the mean ± S.D. of three individual experiments. **P<0.01 compared with RPE cell.

### Overexpression of miR-140-5p inhibits RB cell growth

To investigate the role of miR-140-5p in RB, the Y79 and Weri-Rb1 cells were transfected with miR-140-5p mimics or mimics NC, and the qRT-PCR was used to assess the overexpression efficiency of miR-140-5p. As shown in Figure 2A, miR-140-5p is significantly overexpressed in both Y79 and Weri-Rb1 compared with mimics NC (*P*<0.01). Then, we performed the CCK-8 assay and flow cytometry analysis to measure the cell proliferation and apoptosis in miR-140-5p-overexpressed Y79 and Weri-Rb1 cells, respectively. We found that overexpression of miR-140-5p dramatically suppresses cell proliferation and promotes apoptosis compared with mimics NC (*P*<0.01; Figure 2B–D). Furthermore, flow cytometry analysis further confirmed that overexpression of miR-140-5p led to a marked delay in the ability of arrested cells to progress beyond the G_0_/G_1_ phase block (Figure 2E,F; *P*<0.01). These results indicated that miR-140-5p exerts the suppressive effects on RB cells via inhibiting proliferation and inducing apoptosis and cell cycle arrest.

**Figure 2:** miR-140-5p represses RB cell growth and cell cycle (**A**) The qRT-PCR was used to evaluate overexpression efficiency of miR-140-5p in the Y79 and Weri-Rb1 cells transfected with miR-140-5p mimics or mimics NC. (**B**,**C**) The CCK-8 assay was conducted to determine cell proliferation in the Y79 and Weri-Rb1 cells transfected with miR-140-5p mimics or mimics NC, respectively. (**D**) The cell apoptosis was measured using flow cytometry analysis in the Y79 and Weri-Rb1 cells transfected with miR-140-5p mimics or mimics NC. (**E**,**F**) The flow cytometry analysis was performed to evaluate the cell cycle in the Y79 and Weri-Rb1 cells transfected with miR-140-5p mimics or mimics NC, respectively. Data were presented as the mean ± S.D. of three individual experiments. *P<0.05, **P<0.01 compared with mimics NC.

### *c-Me*t is a target gene of miR-140-5p in RB cells

Mounting studies revealed that miR-140-5p was identified to act as a tumor suppressor in various cancers via suppressing its target gene, such as hypopharyngeal cancer, biliary tract cancer, and gastric cancer [19,20]. In our study, we performed the TargetScan and miRanda to predict the target genes of miR-140-5p, and identified c-Met as a potential target of miR-140-5p (Figure 3A). To validate this bioinformatics predication, the wt or mut type of c-Met-3′-UTR was constructed and inserted into the firefly luciferase expressing vector pMIR-REPORT (Figure 3B). Subsequently, the Y79 cells were co-transfected with wt or mut reporter plasmid along with miR-140-5p mimics/inhibitor or NC, and measured the luciferase activity. As shown in Figure 3C, miR-140-5p mimics markedly inhibited the luciferase activity of the wt-c-Met-3′-UTR compared with mimics NC, whereas miR-140-5p inhibitor significantly enhanced the luciferase activity (*P*<0.01). However, miR-140-5p did not suppress the luciferase activity of the reporter vector binding 3′-UTR of c-Met with mutations in the miR-140-5p-binding site (Figure 3C). To further confirm the c-Met expression is regulated by miR-140-5p, we performed the Western blot assay to detect the c-Met expression in Y79 and Weri-Rb1 cells treated with mimics/inhibitor or NC. We found that overexpression of miR-140-5p decreased the c-Met expression, but down-regulation of miR-140-5p increased the c-Met level in both Y79 and Weri-Rb1 cells compared with vector (Figure 3D). In addition, IHC showed that c-Met level is dramatically up-regulated in RB tissues compared with normal retinas (Figure 3E). To clarify the relationship between miR-140-5p and c-Met in RB, the qRT-PCR assay was used to determine the mRNA level of c-Met in RB tissues (*n*=50). The results illustrated that c-Met expression is obviously increased in the 50 cases of tumors compared with normal retinas (*n*=8) (*P*<0.01; Figure 3F). Correlation analysis also showed a dramatically negative correlation between miR-140-5p level and c-Met expression in 50 tumor tissues (r = −0.8137, *P*<0.01; Figure 3G). Collectively, these results suggested that miR-140-5p negatively regulated c-Met expression and their inversely correlation could be determined in clinical tissues.

**Figure 3:** *c-Met* is a target gene of miR-140-5p in RB cells (**A**) Prediction of c-Met as a target of miR-140-5p in different species. (**B**) Schematic view of miR-140-5p putative targetting site in the wt and mut 3′-UTR of c-Met. (**C**) The relative luciferase activity of c-Met wt or mut 3′-UTR in Y79 cells transfected with the miR-140-5p mimic/inhibitor or corresponding NC. **P<0.01 compared with mimics NC, ^##^*P*<0.01 compared with the inhibitor NC. (**D**) The Western blot analysis was used to detect the protein level of c-Met in the Y79 and Weri-Rb1 cells transfected with miR-140-5p mimics/inhibitor or corresponding NC, respectively. β-actin served as an internal control. **P<0.01 compared with mimics NC, ^##^*P*<0.01 compared with inhibitor NC. (**E**) IHC was used to detect c-Met expression in RB tissues and normal retinas. (**F**) The miR-140-5p was determined by the qRT-PCR in RB tissues (*n*=50) and normal retinas (*n*=8). (**G**) The negative correlation between c-Met and miR-140-5p levels in the RB patients (r = −0.8137, *P*<0.01). Data were presented as the mean ± S.D. of three individual experiments.

### c-Met silencing inhibits RB cell proliferation and induces apoptosis and cell cycle arrest

To further explore the role of c-Met in RB cell, c-Met was inhibited by si-c-Met in Y79 or Weri-Rb1 cells, and then cell viability, apoptosis, and cell cycle were assessed using CCK-8 assay and flow cytometry, respectively. As shown in Figure 4A, the protein and mRNA level of c-Met were markedly down-regulated in Y79 or Weri-Rb1 cells transfected with si-Met when compared with that si-scramble (*P*<0.01). Then, our results demonstrated that c-Met silencing obviously suppressed cell proliferation and promoted apoptosis in both the Y79 and Weri-Rb1 cells compared with si-Scramble (*P*<0.01; Figure 4B,C). As expected, inhibition of c-Met resulted in a marked delay in the ability of arrested cells to progress beyond the G_0_/G_1_ phase block (*P*<0.01; Figure 4D,E). These results suggested that c-Met act as an oncogene through regulating cell proliferation, apoptosis, and cell cycle in RB.

**Figure 4:** c-Met silencing inhibits RB cell proliferation and induces apoptosis and cell cycle arrest The Y79 or Weri-Rb1 cells were transfected with si-c-Met or si-Scramble. (**A**) The protein and mRNA levels of c-Met were evaluated by the Western blot analysis and qPCR analysis. β-actin served as an internal control. (**B**) The CCK-8 assay was used to evaluate cell proliferation in the Y79 and Weri-Rb1 cells. (**C**) The cell apoptosis was determined using flow cytometry analysis. (**D**,**E**) The cell cycle was measured in the Y79 and Weri-Rb1 cells by flow cytometry analysis, respectively. Data were presented as the mean ± S.D. of three individual experiments. **P<0.01 compared with si-Scramble.

### c-Met rescues the suppressive effects of miR-140-5p on RB cell growth and cell cycle arrest

To investigate whether c-Met is a functional target of miR-140-5p, the Y79 or Weri-Rb1 cells were transfected with miR-140-5p mimics/inhibitor or were co-transfected with miR-140-5p mimics and pcDNA-c-Met plasmid. As shown in Figure 5A, overexpression of miR-140-5p attenuates the protein level of c-Met, but pcDNA-c-Met remarkably rescues the suppressive effects of miR-140-5p on c-Met expression. Then, we performed the CCK-8 assay and flow cytometry analysis to evaluate cell proliferation, apoptosis, and cell cycle in each group. The results demonstrated that miR-140-5p significantly inhibited cell proliferation and induced apoptosis and cell cycle arrest, but the suppressive action of miR-140-5p on RB cells were obviously abrogated by c-Met overexpression in both the Y79 and Weri-Rb1 cells (Figure 5B–F). These data indicated that miR-140-5p exerts the suppressive effects on RB cells through modulating c-Met expression.

**Figure 5:** c-Met rescues the effects of miR-140-5p-mediated RB cell proliferation, apoptosis, and cell cycle The Y79 or Weri-Rb1 cells were transfected with miR-140-5p mimics or were co-transfected with miR-140-5p mimics and pcDNA-c-Met. (**A**) The protein level of c-Met was evaluated by the Western blot analysis. β-actin served as an internal control. (**B**,**C**) The CCK-8 assay was used to evaluate cell proliferation in the Y79 and Weri-Rb1 cells, respectively. (**D**) The cell apoptosis was determined using flow cytometry analysis. (**E**,**F**) The cell cycle was measured in the Y79 and Weri-Rb1 cells by flow cytometry analysis, respectively. Data were presented as the mean ± S.D. of three individual experiments. *P<0.05, **P<0.01 compared with mimics NC, ^##^*P*<0.01 compared with miR-140-5p mimics.

### miR-140-5p suppresses c-Met/AKT/mTOR signaling pathway

The PI3K/AKT/mTOR signaling pathway is a key downstream pathway of c-Met, which could modulate various biological processes, including cell proliferation, metastasis, and angiogenesis [21]. Previous study revealed that miR-206 could suppress the PI3K/AKT/mTOR signaling axis via targetting c-Met in non-small cell lung cancer [22]. To investigate whether miR-140-5p inhibit RB cell growth and cycle through modulating c-Met/AKT/mTOR signaling pathway, the Y79 and Weri-Rb1 cells were transfected with miR-140-5p mimics or mimics NC and the p-c-Met, c-Met, p-AKT, AKT, p-mTOR, mTOR, p-S6, and S6 were analyzed by Western blot analysis. We found that overexpression of miR-140-5p significantly attenuated the expression of p-c-Met, p-AKT, p-mTOR, and p-S6 in both Y79 and Weri-Rb1 cells compared with control vector (*P*<0.01; Figure 6A–C). These results indicated that miR-140-5p may act as a tumor suppressor in RB through suppressing c-Met/AKT/mTOR signaling pathway.

**Figure 6:** miR-140-5p suppresses c-Met/AKT/mTOR signaling pathway (**A**) The p-c-Met, c-Met, p-AKT, AKT, p-mTOR, mTOR, p-S6, and S6 were analyzed by Western blot analysis in Y79 cells and Weri-Rb1 cells transfected with miR-140-5p mimics or mimics NC. (**B**,**C**) Quantitative analysis of all proteins expression in Y79 cells and Weri-Rb1 cells transfected with miR-140-5p mimics or mimics NC. β-actin served as an internal control. Data were presented as the mean ± S.D. of three individual experiments. *P<0.05, **P<0.01 compared with mimics NC.

## Discussion

Increasing studies documented that miR-140-5p serves as a tumor suppressor in various types of cancers [13–16]. However, the roles of miR-140-5p in RB remain elusive. In the present study, we demonstrated that miR-140-5p is obviously down-regulated in RB tissues and cells, low miR-140-5p expression is associated with clinicopathological features and poor survival in RB patients. Moreover, our results showed that miR-140-5p suppresses proliferation and induces apoptosis and cell cycle arrest via targetting c-Met. More importantly, our data revealed that miR-140-5p exerts the suppressive effects on RB cell through blocking c-Met/AKT/mTOR signaling pathway.

Many miRNAs have been demonstrated to be associated with RB development and occurrence by regulating and inhibiting the expression of their target gene, and function as oncogene or tumor suppressor [23,24]. Wu et al. uncovered that miR-204 represses RB cell proliferation and invasion by targetting CyclinD2 and MMP-9 [7]. Wang et al. [10] documented that miR-183 suppresses RB cell proliferation, migration, and invasion through down-regulating low-density lipoprotein receptor-related protein 6 (LRP6). Specifically, mounting evidence indicated that miR-140-5p plays the role as a tumor suppressor in many cancers, such as ovarian cancer [14], non-small cell lung cancer [15], colorectal cancer [16], and gastric cancer [13]. However, the potential role of miR-140-5p in RB remains elusive. In the present study, we found that the expression of miR-140-5p in RB tissues and cells are dramatically lower than normal retinas and RPE cells. Moreover, we confirmed that low expression of miR-140-5p significantly correlated with clinicopathological features (differentiation, invasion, T classification, N classification, cTNM stage, and largest tumor base) and poor survival. These results indicated that low miR-140-5p expression predicts poor prognosis in RB, suggesting that miR-140-5p may act as a potential prognostic biomarker for RB.

To further explore the role of miR-140-5p in RB, the Y79 and Weri-Rb1 cells were transfected with miR-140-5p mimics or mimics NC, and cell proliferation, apoptosis, and cell cycle were determined using CCK-8 assay and flow cytometry. Our results demonstrated that overexpression of miR-140-5p dramatically inhibits cell proliferation and induces apoptosis and cell cycle arrest. These data suggested that miR-140-5p may function as a tumor suppressor in RB.

The c-Met receptor tyrosine kinase, which has been identified as a proto-oncogene and is expressed in both normal and malignant cells [25]. c-Met has been considered to play an important role in the cell growth and metastasis of cancer, and up-regulation of c-Met has a key role in tumor development [26,27]. In this study, we confirmed that *c-Met* is a target gene of miR-140-5p in RB cells, and its expression is significantly up-regulated in RB tissues compared with normal retinas. In addition, correlation analysis showed an obviously negative correlation between miR-140-5p and c-Met expression in RB tissues. Importantly, our results demonstrated that the suppressive effects of miR-140-5p on RB cell growth and cycle were rescued by overexpression of c-Met. Moreover, inhibition of c-Met by si-c-Met represses RB cell proliferation and induces apoptosis and cell cycle arrest. Collectively, these data indicated that miR-140-5p suppresses cell proliferation and induces apoptosis and cell cycle arrest in RB via targetting c-Met.

c-Met is the receptor for hepatocyte growth factor (HGF) is a key regulator in cancer cells, such as cell motility, invasion, and metastasis [28]. The HGF/c-Met signaling pathway is a major contributor to invasive growth, its downstream signaling components include the Ras/MAPK, PI3K/AKT, and the JAK/STAT pathway, which could modulate a variety of the biological processes, such as proliferation, scattering/motility, invasion, survival, and angiogenesis [29,30]. It has been reported that miR-206 suppresses HGF-induced epithelial–mesenchymal transition (EMT) and angiogenesis in non-small cell lung cancer through targetting c-Met/PI3k/AKT/mTOR pathway [22]. Inspired by these studies, we speculated whether miR-140-5p could regulate PI3k/AKT/mTOR signaling pathway in RB cell via targetting c-Met. Our results showed that overexpression of miR-140-5p obviously attenuated the expression of p-c-Met, p-AKT, p-mTOR, and p-S6 in RB cells compared with control vector. Taken together, these data suggested that miR-140-5p harbors the suppressive effects on RB cell growth and cell cycle by blocking c-Met/AKT/mTOR signaling pathway.

In summary, we demonstrated that miR-140-5p is obviously down-regulated in RB tissues and cell lines. Moreover, overexpression of miR-140-5p inhibits proliferation and induces apoptosis and cell cycle arrest in RB cells. In addition, we identified that c-Met is the functional target of miR-140-5p in RB cell. Importantly, miR-140-5p possesses the suppressive effects on RB cell via inhibiting c-Met/AKT/mTOR signaling pathway. Our findings suggested that miR-140-5p may serve as a potential biomarker for prognosis and a therapeutic target for RB patients.

## Abbreviations

Akt: protein kinase B
CCK-8: cell counting kit-8
c-Met: cellular mesenchymal-epithelial transition factor
cTNM: clinical TNM staging
GAPDH: glyceraldehyde‐3‐phosphate dehydrogenase
HGF: hepatocyte growth factor
HRP: horseradish peroxidase–conjugated
IHC: immunohistochemistry
JAK/STAT: Janus kinase/signal transduction and activator of transcription
MAPK: mitogen-activated protein kinase
MMP-9: matrix metalloproteinase-9
mut: mutant
mTOR: mammalian TOR
NC: negative control
PI3K: phosphoinositide 3-kinase
qRT-PCR: quantitative reverse transcriptase PCR
RAS: renin-angiotensin system
RB: retinoblastoma
RPE: retinal pigment epithelium
RT-PCR: reverse transcription PCR
U6: small nuclear RNA U6
wt: wild-type
